# Three-Dimensional Reconstruction of a CT Image under Deep Learning Algorithm to Evaluate the Application of Percutaneous Kyphoplasty in Osteoporotic Thoracolumbar Compression Fractures

**DOI:** 10.1155/2022/9107021

**Published:** 2022-04-28

**Authors:** Jiameng Li, Zhong Xiang, Jiaqing Zhou, Meng Zhang

**Affiliations:** Department of Spine Surgery, The Fourth Hospital of Changsha, Changsha 412002, Hunan, China

## Abstract

In order to investigate the therapeutic evaluation of percutaneous kyphoplasty (PKP) for the treatment of osteoporotic thoracolumbar compression fractures by three-dimensional (3D) reconstruction of computed tomography (CT) based on the deep learning V-Net network, the traditional V-Net was optimized first and a new and improved V-Net was proposed. The introduced U-Net, V-Net, and convolutional neural network (CNN) were compared in this study. Then, 106 patients with osteoporotic thoracolumbar compression fractures were enrolled, and 128 centrums were divided into the test group with 53 cases of PKP and the control group with 53 cases of percutaneous vertebroplasty (PVP) according to different surgical protocols. All patients underwent CT scan based on the improved V-Net, and data of centrum measurement indicators, pain score, and therapeutic evaluation results of the modified Macnab were collected. The Dice coefficient of the improved V-Net was observably higher than that of U-Net, V-Net, and CNN, while the Hausdorff distance was lower than that of U-Net, V-Net, and CNN (*P* < 0.05). The anterior height, central height, and posterior height of the centrum were significantly higher than those in the control group after operation (3, 5, and 7 days), while the Cobb angle of vertebral kyphosis was significantly lower than that in the control group (*P* < 0.05). The score of visual analog scale (VAS) and analgesic use score of patients in the test group were markedly lower than those in the control group (3, 5, and 7 days after operation), *P* < 0.05. Besides, the excellent and good rate of the test group was remarkably higher than that of the control group, *P* < 0.05. Hence, the improved V-Net had better quality of segmentation and reconstruction than the traditional deep learning network. Compared with PVP, PKP was helpful in restoring the height of the centrum in patients with osteoporotic thoracolumbar compression fractures and correct kyphosis, with better analgesic effect safety.

## 1. Introduction

With the increasing aging of population in China, the incidence of osteoporosis in the elderly is increasing. Osteoporotic vertebral fracture is one of the most pervasive complications of osteoporosis [1, 2]. Most patients have no obvious trauma or only mild trauma, such as sprains, bumps, flat falls, and even coughing, sneezing, bending, and other daily movements, which cause fractures easily, with a very high prevalence rate, higher than the hip, wrist, and proximal humerus fractures combined [3–5]. The main clinical symptoms of osteoporotic vertebral fracture are acute or chronic persistent pain in the lower back, chest and back, and chest and rib. The pain is relieved when patients lie down and have a rest but is intensified during activities with muscle convulsions and other phenomena simultaneously [6, 7]. Therefore, vertebral fractures are most common at the thoracolumbar junction and in the middle thoracic vertebrae. Moreover, conservative or surgical treatment is generally carried out according to the degree of patient's condition [8]. There are many conservative treatment methods, however, this treatment takes a quite long time to recovery. Besides, surgical treatment includes percutaneous kyphoplasty (PKP) and percutaneous vertebroplasty (PVP), both of which have such advantages as simple operation, less trauma, and fewer complications [9, 10].

With the pervasiveness of computer technology and imaging, the imaging technology is used in the clinical examination of orthopedic diseases. X-ray, as the most traditional imaging technology, is widely used and helps to show the status of vertebral fractures clearly, but it is prone to misdiagnose and missed diagnosis [11, 12]. The fracture condition is determined by magnetic resonance imaging (MRI) through a multiparameter condition and multiple signals, so MRI has high sensitivity and accuracy. However, MRI is expensive with complex operation, so it is not suitable for frequent use. Both computed tomography (CT) imaging and conventional X-ray use the principle of X-ray to diagnose the conditions of fracture effectively, whose operation is relatively simple and cost is acceptable [13]. Clinically, deep learning technology is often introduced to process original images to help doctors assess patients' conditions more precisely in order to improve the quality of the image [14, 15]. Deep learning is a set of algorithms that use various machine learning algorithms to solve various problems, such as images and texts on multilayer neural networks, which can be regarded as the most mainstream artificial intelligence (AI) at present. Furthermore, one of the hot topics of current research studies is the combinations of deep learning with clinical medical imaging [16]. Therefore, the 3D reconstruction model of CT imaging based on deep learning technology was explored to offer help for image evaluation of orthopedic diseases.

To sum up, osteoporotic vertebral fracture is a major clinical problem in the elderly. Surgical treatment is still advocated. Further studies are needed to evaluate the efficacy and safety of different surgeries. Therefore, traditional V-Net was optimized, and a new and improved V-Net was proposed in the study. The new and improved V-Net was used to scan CT images of 106 patients with osteoporotic thoracolumbar compression fractures who underwent PVP or PKP operation. Vertebral body measurements, pain scores, and efficacy assessment results of the modified Macnab were compared between test group and control group to investigate the clinical effect of PKP and PVP in the treatment of osteoporotic thoracolumbar compression fracture, which could provide some reference for clinical work of osteoporotic thoracolumbar compression fractures.

## 2. Materials and Methods

### 2.1. Subjects of the Study

One hundred six patients with osteoporotic thoracic and lumbar compression fractures who underwent PVP or PKP operation in hospital from June 1, 2018, to November 30, 2021, were included in the study. There were 128 centrums, including 63 males and 43 females. In accordance with the different surgical programs, the patients were divided into the test group with 53 cases of PKP and the control group with 53 cases of PVP. All the patients volunteered to participate and signed informed consent prior to the implementation of the study. This study had been approved by the ethics committee of the hospital.

The inclusion criteria were as follows: (I) patients diagnosed with severe osteoporosis by routine examination; (II) patients with intact posterior wall of centrums; (III) patients without the symptoms of spinal cord injury; and (IV) patients without the symptoms of nerve root damage.

The exclusion criteria were as follows: (I) patients with a compression fracture caused by a hemangioma; (II) patients with a compression fracture due to vertebral metastases; (III) patients with contraindications for operation; (IV) patients with poor compliance; and (V) patients with incomplete clinical data.

### 2.2. Therapeutic Schedule

Patients in the test group were placed in the supine position with pads placed on both sides of the hip. A unilateral pedicle approach was used to locate the responsible centrum with the X-rays on the C-arm machine and Kirschner wire (K-wire). Then, the projection of the pedicle to the transverse process was inserted with a puncture needle. When it reached the middle of the centrum, the puncture needle was immediately pulled out, the guide needle was inserted, and the prepared bone cement was slowly injected into the centrum. Meanwhile, CT was used to observe the distribution of bone cement. Additionally, after the distribution of bone cement was satisfied, the injection was stopped and hemostasis was performed. Antibiotics were applied 1-2 days after the operation. The patient was put on braces for activities 1 day later.

Patients in control group were placed in the supine position with pads placed on both sides of the hip. A unilateral pedicle approach was used to locate the responsible centrum with the X-rays on the C-arm machine and K-wire. Next, a puncture needle was placed in the line between the pedicle projection and the transverse process. When the middle of the centrum was reached, the needle was pulled out and a guide one was inserted. Along the guide needle, expansion casing and working casing were placed, and the fine drill was screwed in. After the fine drill was close to the anterior edge of the centrum, the drill was pulled out, and the pressurized balloon was put into the centrum. Then, the contrast agent was injected into the pressurized balloon with a syringe, and when the reduction was satisfactory, the injection was stopped. The contrast agent was pumped back and the balloon was pulled out. The prepared bone cement was slowly injected into the centrums. Meanwhile, the distribution of bone cement was observed by CT. The injection was stopped and hemostasis was performed after the distribution was satisfied. Antibiotics were applied one or two days after the operation. Additionally, patients were asked to put on braces for activities 1 day later.

### 2.3. Examination of CT Imaging

128 slice spiral CT was used. Patients were asked to be in the supine position. The scan area was each centrum in the horizontal direction of the suspected injury, so that the scanning plane was perpendicular to the spinal canal. The parameters were set as follows: layer thickness was 0.521 mm, layer spacing was 1.2 mm, scanning dose was 120 kV, 250 mass, and measuring distance accuracy was 0.15 mm.

Then, the images obtained were transmitted to the workstation. After treatment, the leading edge, trailing edge, central height, and kyphosis Cobb angle of responsible centrums were measured.

### 2.4. Improved V-Net

The neural network is a mathematical model or computational model that imitates the structure and function of the biological neural network, which consists of the input layer, hidden layer, and output layer. As a technology oriented to 3D data processing, V-Net neural network [17] belongs to the coding-decoding structure. Moreover, the network on the left continuously helps to reduce the resolution of the image to extract features, and the right one is helpful to decode the image to restore it to the original size. A new V-Net based on the optimization of traditional V-Net is proposed in this study (Figure 1). The whole network structure is classified into the left side and the right side. The left side is the data compression part, and the right one is the data expansion part. Besides, each side has three feature channels, the input module is 120 × 120 × 56, and the up-down sampling convolution kernel is 2 × 2 × 2.

The activation function of convolution postsampling is parametric rectified linear unit (PReLU) function.

The function is as follows:

(1) $$\begin{array}{c} \text{ReLU}\left(x\right)=\left\{\begin{array}{cc} 0, & x\geq 0,\\ x, & x<0. \end{array}\right.. \end{array}$$

When *x* < 0, the ReLU function is hard saturated. When *x*=0, there is no saturation problem in the ReLU function. When *x* > 0, the ReLU function is not exhausted, and the gradient problem is solved. The ReLU function is improved to solve the problem of hard saturation, and the PReLU function is obtained, as shown in

(2) $$\begin{array}{c} \text{PReLU}\left(x\right)=\left\{\begin{array}{cc} 0, & x\geq 0,\\ x, & \beta x<0. \end{array}\right.. \end{array}$$

In (2), *β* is a learnable parameter, not a fixed value. Then, the Softmax classifier is used to calculate the probability of the category of image pixels, as shown in

(3) $$\begin{array}{c} G\left(j\right)=\frac{e^{x_{j}}}{\sum_{j=1}^{M}e^{x_{j}}}. \end{array}$$

In the (3), *G*(*j*) represents the probability value that the pixel belongs to the j-th class, and *x*_*j*_ represents the j-th value in a pixel feature vector. The category corresponding to the maximum probability of each pixel is the category of the pixel, thus obtaining the final semantic segmentation result.

### 2.5. Evaluation Indicators

U-Net [18], V-Net, and CNN [19] were introduced for comparative analysis with the optimized V-Net designed in this study. The Dice coefficient, Hausdorff distance, and other indicators were used to evaluate the segmentation and reconstruction consequences of images by each deep learning network.

(4) $$\begin{array}{c} \text{Dice}=\frac{2\times \left|Z_{1}\cap Z_{2}\right|}{\left|Z_{1}\right|+\left|Z_{2}\right|},\\ \text{Hausdorff}=\max\left(\text{Hausdorff}\left(C_{1},C_{2}\right),\text{Hausdorff}\left(C_{2},C_{1}\right)\right),\\ \text{Hausdorff}\left(C_{1},C_{2}\right)=\max_{c_{1}\in C_{1}}\min_{c_{2}\in C_{2}}\left\|c_{1}-c_{2}\right\|,\\ \text{Hausdorff}\left(C_{2},C_{1}\right)=\max_{c_{2}\in C_{2}}\min_{c_{1}\in C_{1}}\left\|c_{2}-c_{1}\right\|. \end{array}$$

In the abovementioned functions, *Z*_1_ represented the actual result, *Z*_2_ represented the segmentation results, and |⋯| represented all the pixel value. *C*_1_ and *C*_2_ represented the two sets. Hausdorff(*C*_1_, *C*_2_) represented the unidirectional Hausdorff distance from *C*_1_ to *C*_2_, and Hausdorff(*C*_2_, *C*_1_) represented the unidirectional Hausdorff distance from *C*_2_ to *C*_1_.

### 2.6. Therapeutic Evaluation

The visual analog scale (VAS), analgesic use score, and activity ability score of the patients were recorded before operation, and at 3, 5, and 7 days after operation. The modified Macnab was used to grade and evaluate the postoperative recovery of patients (excellent, good, medium, and poor).

### 2.7. Statistical Methods

SPSS 19.0 was employed for data statistics and analysis. Mean±standard deviation (*x̄* ± *s*) was how measurement data were expressed. The enumeration data were expressed in percentage. One-way analysis of variance was employed for pairwise comparison. When *P* < 0.05, it meant that the difference was statistically significant.

## 3. Results

### 3.1. Clinical Data of Patients

Figure 2 shows that there were no significant differences in sex ratio, symptom duration, the number of centrums (T8-T12 and L1-L5), age, height, and weight between test group and control group, *P* > 0.05.

### 3.2. Medical Records of Some Patients

Figures 3 and 4 show preoperative and postoperative CT images of different patients. The distribution of the fractured centrums was shown clearly through the preoperative CT images. The distribution of bone cement in centrums was shown through the postoperative CT images. Additionally, the centrums were fully filled with bone cement and the position of vertebral fracture was repaired.

### 3.3. Performance Comparison of Different Deep Learning Networks

In Figure 5, the Dice coefficient of the improved V-Net in this study was markedly higher than that of U-Net, V-Net, and CNN (*P* < 0.05). Furthermore, the Hausdorff distance of the improved V-Net was significantly lower than that of U-Net, V-Net, and CNN (*P* < 0.05).  Figure 6 shows the spine 3D reconstruction images of the improved V-Net, where this deep learning network had a fabulous impact on 3D reconstruction of CT images, which completely constructed the spine structure and retained good details.

### 3.4. Vertebral Imaging Results of the Two Groups

In Figure 7, before the operation, there were no statistically significant differences in vertebral anterior height, central height, posterior height, and kyphosis Cobb angle between the two groups. The anterior height, central height, and posterior height of centrums in test group were greatly higher than those in control group (*P* < 0.05). Besides, after the operation (3, 5, and 7 days), the Cobb angle of kyphosis of test group was observably smaller than that of control group (*P* < 0.05).

### 3.5. Comparison of the Scores of the Two Groups before and after Operation

In Figure 8, there were no significant differences in the preoperative VAS score, analgesic use score, and ability of activity score in both test group and control group, *P* > 0.05. At 3, 5, and 7 days after operation, the VAS score and analgesic use score of patients in test group were evidently lower than those in control group, *P* < 0.05. Additionally, there was no statistically significant difference in activity scores between the two groups at 3, 5, and 7 days after operation.

### 3.6. Results of Postoperative Efficacy Evaluation of Modified Macnab in Two Groups

Figure 9 shows that there were 33 excellent cases, 13 good cases, 5 medium cases, and 2 poor cases of the modified Macnab in the test group. In the control group, there were 24 excellent cases, 17 good cases, 7 medium cases, and 5 poor cases. Therefore, the excellent and good rate of the test group was obviously higher than that of the control group (*P* < 0.05).

## 4. Discussion

Osteoporosis is a systemic disease of bone metabolism. The main manifestations were the increased bone brittleness, decreased elasticity, and decreased bone density. Osteoporotic vertebral compression fractures can seriously affect the patients' living quality and exercise ability, which requires aggressive rehabilitation [20, 21]. Deep learning combined with CT imaging technology is applied in the diagnosis and treatment of orthopedic diseases. Hence, the traditional V-Net was optimized first in the study. Then, a new improved V-Net was proposed. U-Net, V-Net, and CNN were introduced for comparison. The Dice coefficient of the improved V-Net was remarkably higher than that of V-Net, V-Net, and CNN. However, the Hausdorff distance was notably lower than that of U-Net, V-Net, and CNN, *P* < 0.05. The results were similar to the results of Kyriakou et al. (2019) [22]. Both the Dice coefficient and Hausdorff distance were effective indicators to evaluate the accuracy of image reconstruction. Therefore, the improve V-Net in this study had better segmentation and reconstruction quality than traditional deep learning network [23]. According to the 3D reconstruction results, the improved V-Net had excellent impacts of 3D reconstruction on CT images. Besides, it also constructed the spine structure and retained good details, which was consistent with the above quantities data.

106 patients with osteoporotic thoracolumbar compression fractures were selected. 128 centrums were divided into test group with 53 cases of PKP and control group with 53 cases of PVP. The clinical indicators of the two groups were recorded before and after operation. The anterior height, central height, and posterior height of centrums in test group were markedly higher than those in control group at 3, 5, and 7 days after operation. The Cobb angle of vertebral kyphosis was significantly lower than that in control group, *P* < 0.05. The consequences showed that compared with PVP, PKP treatment was helpful to restore the height of patients' diseased centrums effectively and correct kyphosis [24]. Moreover, at 3, 5, and 7 days after operation, the VAS score and analgesic use score of patients in test group were evidently lower than those in control group, *P* < 0.05. The consequences meant that compared with PVP, PKP treatment had more effective analgesic impact and safety, which was a safely and availably ideal method for the treatment of osteoporotic vertebral compression fracture. Additionally, there were no statistically significant differences in the scores of activity ability between test group and control group at 3, 5, and 7 days after operation, *P* > 0.05. Such results were quietly different from the previous studies. The reason probably was that the sample size included in this study was small, which caused the difference in activity ability between the two groups not obvious [25]. Finally, the modified Macnab was employed to evaluate the postoperative efficacy of the patients, and excellent and good rate of test group was greatly higher than that of control group (*P* < 0.05). The results showed that PKP was more effective than PVP in the treatment of osteoporotic vertebral compression fractures.

## 5. Conclusions

The treatments of PKP and PVP were given to patients with osteoporotic thoracolumbar compression fractures in the experimental group and the control group, respectively. The CT image scanning based on the improved V-Net was performed on all the patients. Comprehensive evaluation results showed that PKP had a definite efficacy, analgesic effect, and good safety in patients with osteoporotic thoracolumbar compression fractures. The deficiency of this experiment is that the sample size of included patients is too small, which is limited to patients with thoracolumbar compression fractures. Moreover, the performance analysis of the improved V-NET network is not sufficient. A large number of data set samples are required for verification. The in-depth analysis will be considered later. In conclusion, the results of this study provided help for the clinical adoption of deep learning technology combined with imaging, which had a certain reference value for the clinical work of osteoporotic thoracolumbar compression fractures.

## Figures and Tables

**Figure 1:** Structure of the improved V-Net.

**Figure 2:** Clinical data of patients. (a) Sex ratio and symptom duration. (b) Number of centrums (T8-T12 and L1-L5). (c) Age, height, and weight.

**Figure 3:** 70-year-old female with compression fractures of thoracic 12 and lumbar 1 vertebral body. (a) Preoperative CT. (b, c) Postoperative CT of thoracic 12 and lumbar 1 vertebral body.

**Figure 4:** 73-year-old female with a compression fracture of the first lumbar vertebra. (a) Preoperative CT. (b) Postoperative CT of lumbar 1 vertebral body.

**Figure 5:** Comparison of the Dice coefficient and Hausdorff distance of different deep learning networks. Compared with the improved V-Net in this study, *P* < 0.05.

**Figure 6:** 3D reconstruction images of spine in the improved V-Net.

**Figure 7:** Vertebral imaging results of the two groups. (a) Anterior height, (b) central height, (c) posterior height, and (d) kyphosis Cobb angle, respectively. Besides, the numbers 0, 3, 5, and 7 meant before operation and 3, 5, and 7 days after operation, respectively. Compared with the test group, *P* < 0.05.

**Figure 8:** Comparison of preoperative and postoperative scores between the two groups. The numbers, 0, 3, 5, and 7 meant before operation and 3, 5, and 7 days after operation, respectively. (a) VAS score. (b) Analgesic use score. (c) Ability of activity score. ^*∗*^Compared with the test group, *P* < 0.05.

**Figure 9:** Comparison of postoperative adverse event between the two groups. (a) Number of the difference among the number of excellent, good, medium, and poor cases. (b) Excellent rate. *∗*Compared with the high-intensity group, *P* < 0.05.

## Data Availability

The data used to support the findings of this study are available from the corresponding author upon request.
